The article "The Efficiency of AuNPs in Cancer Cell Targeting Compared to Other Nanomedicine Technologies Using Fuzzy PROMETHEE" was published in 2021. Journal: J Healthc Eng.

# The Efficiency of AuNPs in Cancer Cell Targeting Compared to Other Nanomedicine Technologies Using Fuzzy PROMETHEE

**DOI:** 10.1155/2021/1566834

**Published:** 2021-09-15

**Authors:** Safa Anmar Albarwary, Ayse Gunay Kibarer, Mubarak Taiwo Mustapha, Hani Hamdan, Dilber Uzun Ozsahin

**Affiliations:** ^1^Department of Biomedical Engineering, Innovation and Information Technologies Center, Near East University, Nicosia, Cyprus; ^2^Department of Mechatronics, Tishk International University, Erbil, Iraq; ^3^DESAM Institute, Near East University, Nicosia, Turkish Republic of Northern Cyprus, Turkey; ^4^Université Paris-Saclay, CNRS, CentraleSupélec, Laboratoire des Signaux et Systèmes L2S UMR CNRS 8506, Paris, France; ^5^Medical Diagnostic Imaging Department, College of Health Science, University of Sharjah, Sharjah, UAE

## Abstract

*Cancer* is a disease with rare, diverse symptoms, causing abnormal cell growth in an uncontrolled way, leading to cell damage, apoptosis, and eventually death of the patient. This study uses the Fuzzy PROMETHEE technique to develop a new path for cancer treatment based on nanoparticles (NPs) applications, used in controlled anticancer drug delivery (drug release, toxicity, and unspecific site targeting) to enhance patient safety. The different nanoparticles employed in the drug delivery analysis are gold nanoparticles (AuNPs), liposomes, dendrimers, polymeric micelles (PMs), and quantum dots (QDs). Fuzzy predictable preference organization mode and evaluation multicriteria choice were used as tactics in making the best decision using the data from the factors of cost, size, shape, surface charge, ligand type, pH and temperature stimuli, biocompatibility, accumulation ratio, toxicity, specificity, stability, efficacy, adverse effect, and safety factor of the NPs. The results obtained from the total net flow of the visual PROMETHEE scenario for anticancer drug delivery, based on NPs data analysis, show that AuNPs are ranked the highest among the other NPs. The Phi values obtained for the NPs are as follows: AuNPs (0.1428), PMs (0.0280), QDs (−0.0467), dendrimers (−0.0593), and liposomes (−0.0649). This study highlights the optimal choice of NPs as an intelligent drug delivery system that facilitates therapeutic efficiency, where cancer cells are accurately targeted to enhance treatment quality and patient safety.

## 1. Introduction

Cancer is a disease with rare, diverse symptoms, causing abnormal cell growth in an uncontrolled way, leading to cell damage, apoptosis, and eventually death of the patient [1]. In the United States, an estimation made by the American Society of Cancer found the estimated data of new cancer incidence. Their report shows that no fewer than 1,762,450 new cancer cases were recorded in 2019, while 606,880 mortality cases were recorded [2]. Moreover, there have been projections of the number of new cases of cancer for the next decades. One of such projections was made by the World Health Organization (WHO). The global health body WHO estimated that in 2018 cancer accounted for about 9.6 million deaths globally [3, 4], with the deaths projected to reach up to 22 million by the year 2035. This shows the rate at which cancer is increasing, and how important it is to contribute to fighting it.

The article "The Efficiency of AuNPs in Cancer Cell Targeting Compared to Other Nanomedicine Technologies Using Fuzzy PROMETHEE" was published in 2021. Journal: J Healthc Eng.

Different cancer treatment techniques are used alternatively. This includes surgery, chemotherapy, and radiotherapy. Chemotherapy is the most widely used technique to eliminate tumors and cancer cells. However, the chemotherapy technique usually lacks efficacy on the specificity of targeting cancer cells without harming nearby healthy cells or tissues. This is harmful to the patient and may result in several side effects that may be active throughout the patient's lifespan. Therefore, the need to increase the efficacy of chemotherapy and other cancer therapies is necessary to reduce the severity and adverse side effects of these treatment techniques. The classical anticancer drugs are characterized by poor control of the drug-releasing process and biodistribution in the body of the patient. Other characteristics include low effectiveness and unspecific selectivity with undesirable adverse side effects. To improve the efficiency of the drug delivery process for the targeted site, there is a need to deliver fewer doses of these anticancer drugs to achieve fewer undesirable side effects.

One promising technique to improve the efficiency of the anticancer drug in targeted sites is nanoparticles (NPs). NPs are considered one of the most attractive choices in targeting and killing cancer cells with significantly reduced side effects. They can behave with highly flexible biological properties offered by their extra small size, between 1 and 100 nm, and high surface to area ratio. These excellent characteristics give NPs the ability to be linked and adsorbed with anticancer drug delivery agents at a wide range of modulation to improve high efficacy. Problems associated with uncontrollable drug delivery to desired targeted sites are not new. However, NPs are used as a control agent in the drug delivery process to reach desired targeted sites. According to [5], nanodrug delivery system protects against rapid degradation and enhances drug concentration in target tissues. This smart drug delivery system can be achieved by engineering the surface features of nanoparticles to enhance biocompatibility, stability, efficacy, and patient's safety [6].

The article "The Efficiency of AuNPs in Cancer Cell Targeting Compared to Other Nanomedicine Technologies Using Fuzzy PROMETHEE" was published in 2021. Journal: J Healthc Eng.

Funkhouser first referred to nanotheranostics as a novel technique with the capabilities of simultaneously providing diagnosis and therapy in 2002 [7]. In the last two decades, many studies have been carried out to exploit and develop the unique properties of nanotheranostic agents for cancer treatment. These studies were mainly concentrated on imaging, diagnosis, and treatment. NPs attracted considerable attention in therapy due to weaknesses in classical anticancer drugs. There is also the challenge of choosing the right combination of theranostic agents for accurate cancer cell targeting. About 12,000 research papers have been published on NPs as anticancer drug delivery system, leading to rapid development in this field [8]. The development of NPs for targeted drug delivery is divided into three generations: The first generation focused on the chemistry of the surface particles and main charges to improve biocompatibility and limiting toxicity [9]. The second generation incorporated biocompatible polymers to improve functional properties (e.g., polyethylene glycol (PEG)). This prolongs NPs in blood circulation [10]. Lastly, the third generation focused on developing environmental responsive polymer (e.g., pH and temperature changes), to improve drug delivery efficacy [11].

This study explored a new decision-making process for the selection and combination of the abovementioned three generations with the best specific group of NPs used in cancer therapy. The method used in realizing this aim is the incorporation of fuzzy logic and multicriteria decision-making technique (MCDM) called fuzzy PROMETHEE. Accordingly, a comparative evaluation and ranking of NPs were achieved using several important factors affecting the performance of NPs. These factors included size, shape, surface charge, ligand type, and other important factors that make NPs smart anticancer drug carriers. The main aim is to find the best alternative to improve stability, specificity, and efficacy of cancer therapies and patient's safety enhancement.

### 1.1. Gold Nanoparticles (AuNPs)

Gold nanoparticles (AuNPs) are inorganic nanostructures on the scale of colloidal nanocarriers. They are very resilient nanoparticles due to their unique physical, chemical, electronic, optical, sensing, and biomedical features which make them excellent for use in diverse biomedical fields including cancer theranostics, drug delivery, molecular imaging, and biosensing [12]. Manufacturing AuNPs is easy compared to other NPs. Special properties of AuNPs include flexibility in the desired shape and small size, a very high surface-volume ratio (about 5 nm/20%; 1 nm/100%), and excellent biocompatibility. Consequently, surfaces of AuNPs can be functionalized with covalent or noncovalent bonds in presence of negative charge [13, 14]. Additionally, AuNPs have gotten more attention in academia (anticancer drug delivery) because they are easily designed in a spherical shape, specific tunable size range (1–10 nm) for drug delivery, and long-lasting blood circulation time, with the possibility of exertion with urine and nonsystematic toxicity [15]. AuNPs are the most stable drug carriers with controlled dispersion and regimented drug release with high specificity for the cancer cell site [11–19]. Lastly, AuNPs have minor noncovalent modifications and carry various drug molecules with high capacity, control, and release through internal stimuli (pH and temperature) or external stimuli (light) changes.

The article "The Efficiency of AuNPs in Cancer Cell Targeting Compared to Other Nanomedicine Technologies Using Fuzzy PROMETHEE" was published in 2021. Journal: J Healthc Eng.

AuNPs are potentially useful in different fields of application. The relative stable ligand-gold binding outside the cell and the reduced stability in the cells contribute partly to making golden nanoparticles a good candidate for drug delivery and drug release due to the high intracellular concentrations of glutathione [20]. On-site and real-time metal ion monitoring using AuNPs can be also employed in environmental biology and clinical toxicity [21, 22]. These metals include mercury (Hg^2+^), cadmium (Cd^2+^), lead (Pb^2+^), and cupric ion (Cu^2+^). Glucose has been widely utilized as a clinical indicator of diabetes and has recently earned increasing interest in the analytical biochemistry areas as a whole [23–26]. To date, electrochemical approaches have been regarded as useful for sensing glucose due to the possibility of achieving a better sensitivity of detection. The majority of electrochemical methods utilize the enzyme glucose oxidase (GOx), which catalyzes the oxidation of D-glucose to gluconolactone and the reduction of oxygen to hydrogen peroxide selectively. Because the association between the amino and cysteine groups of proteins and AuNPs is as strong as that of routinely employed thiols, AuNPs make ideal biocompatible surfaces for the immobilization of enzymes and proteins. As a result, amino acids and proteins can be directly adsorbed on AuNPs without any modification at all [27, 28]. The majority of research on biosensors with AuNPs has focused on enzyme electrodes [29, 30]. The application of AuNPs to protein analysis/detection is also an exciting area of research. AuNPs/protein conjugates have found growing use as bioanalytical, diagnostic, and/or immunohistochemical probes throughout the last decade.

The methodologies for synthesizing AuNPs have been constantly changing. Chemists now have a robust toolbox for functionalizing AuNPs by the attachment of various chemicals and biomolecules to the surface of AuNPs, including small molecules, surfactants, dendrimers, polymers, and proteins. Nanoparticles can be easily functionalized with a number of ligands by several techniques, including thiol (−SH) [31], hydroxyl (−OH) [32], phosphine (−PH2) [33], and amine (−NH2) [34]. These functionalized AuNPs exhibit the predicted reactivity and optical, electrical, and biocompatible features. Three extensively used ways for synthesizing AuNPs probes are electrostatic contact, specific recognition (e.g., antibody-antigen, biotin-avidin), and covalent coupling (Au–S bonding).

The article "The Efficiency of AuNPs in Cancer Cell Targeting Compared to Other Nanomedicine Technologies Using Fuzzy PROMETHEE" was published in 2021. Journal: J Healthc Eng.

### 1.2. Liposomes

Liposomes are phospholipid bilayer nanocarriers. They differ in size from 20 nm to many microns with spherical shape. Liposomes consist of cell membrane which is a phospholipid, making up the lipid tail of fatty acid, cholesterol, and polar head group. Gregory Gregordians was the first to show that phospholipids have self-assembled bilayer vehicles when immersed in water [18]. Unmodified liposomes have problems such as instability, drug loading, fast drug release, and short circulation blood time. In anticancer drug delivery, liposomes have difficulties—controlled distribution, toxicity, and removal from the body [8]. However, functionalized liposomes overcome these problems. Liposomes have many advantages as nanovehicles for drug delivery purpose. They prevent undesirable exposure of drug, protect degradation [35], and can distinguish between healthy and cancerous cells using various types of bonds to activate liposomes to target cancer cells [36]. Liposomes can be stimulated by many factors such as pH, temperature change, or light [37]. Liposomes are more biocompatible than other synthetic materials due to their structure. Additionally, other liposomes that have been modified in desired size, shape, and surface functions can control efficacy and toxicity, changes in absorbance, and biodistribution, thus delivering and releasing the drug most desirably. They also decrease their adverse effects when the drug begins to accumulate within the body, prolonging the time in blood circulation and enhancing the duration of action. Nanotheranostic liposomes can carry both diagnostic and therapeutic agents which improve their progress during drug delivery, making them more promising as anticancer theranostic agents [38, 39].

### 1.3. Dendrimers

Dendrimers are a synthetic class of polymers that self-assemble into highly branched 3D controlled spherical structures, with nanosize scale (1–100 nm). Dendrimers have three sections: core, branches, and exterior surface with functional surface groups [40]. The active groups on the surface of dendrimers give a high level of surface functionality and tune the physicochemical features. Furthermore, because of their high biocompatibility, adsorption, and monodisperse nature, they can be used in drug delivery with a higher drug encapsulation rate [41]. Dendrimers can be utilized as anticancer drug delivery and diagnostic agents [42, 43]. For drug delivery, dendrimers can encapsulate drug molecules covalently or noncovalently, depending on whether the drug is encapsulated inside or linked on the dendrimer surface. However, covalent bonds are undoubtedly more stable [44, 45]. Drug leakage, immunogenicity, and cytotoxicity limit the use of dendrimers. They usually have nonspecific drug release, which causes undesired adverse effect and poor efficacy [46]. Though dendrimers can improve polymer accumulation at a specific targeted site and bind to other molecules to adjust solubility, they still have difficulty in controlled drug release at the targeted site [47].

The article "The Efficiency of AuNPs in Cancer Cell Targeting Compared to Other Nanomedicine Technologies Using Fuzzy PROMETHEE" was published in 2021. Journal: J Healthc Eng.

### 1.4. Polymeric Micelles

Polymeric micelles are self-assembled amphiphilic block copolymers. They can be created at specific critical micelle concentration [17]. Polymeric micelles are spherical core-shell structures with nanosizes ranging from 10 to 100 nm. It has been proven that polymeric micelles are an excellent drug delivery system due to their high stability in physiological conditions [5]. Their advantages include their unique size and shape, solubility, drug release at the targeted site, protection of drugs from degradation, surface functionalization's property, and their ability to be modified to decrease toxicity ratio, increase targeting specificity, and improve efficacy, which makes them a proper choice for anticancer drug delivery purposes [48]. The drugs can be loaded into a polymeric micelle physically, chemically, or through electrostatic interactions [49]. Micelles may face undesirable interaction with blood and damage the balance between micelle and blood, besides the undesirable drug release bypassing the “critical micelle concentration.” To overcome this problem, it is necessary to modify polymeric micelles [49, 50]. Many types of bonds and stimuli factors are used to functionalize the polymeric micelles to release the drugs at the desired dose and site [51]. The codelivery technique in the multifunctional micelle is an important factor to the improvement of their effects in cancer treatment and diagnosis [52].

### 1.5. Quantum Dots

Quantum dots (QDs) are nanocrystal inorganic NPs with spherical core-shell structure and nanosize (2–10 nm), consisting of a semiconductor inorganic core and an aquatic organic shell. Their unique features come from their physical nanosize, bright high photostability, and wide range of excitation using UV light [18]. QDs have been modified to achieve a longer time in the intracellular process for bioimaging and monitoring in real time in vitro. They are very useful in the medical field especially as diagnostic agents such as MRI and tissue fluorescence imaging agent, in cell labeling, and for therapeutic purpose in cancer treatment [53]. In an in vitro study, prostate cancer was developed in experimental mice, and QDs have been used as anticancer drug delivery. It was proven that QDs accumulated at cancer sites successfully by promoting permeability and retention effect. To increase the accumulation ratio at the cancer sites, QDs were modified with specific functionalization factors and bonds [54]. However, QDs have critical problems with nonexertion with urine, deposition in lungs, and atriums of the heart, which causes toxicities. The studies and reports on the excretion of QDs are very limited making their clinical usage very difficult [5].

The article "The Efficiency of AuNPs in Cancer Cell Targeting Compared to Other Nanomedicine Technologies Using Fuzzy PROMETHEE" was published in 2021. Journal: J Healthc Eng.

This study investigates the weaknesses of current cancer therapy techniques and how rapid development in nanotechnology is strengthening them. We applied the fuzzy PROMETHEE method to compare dominant criteria of NPs in anticancer drug delivery.

## 2. Materials and Methods

### 2.1. Fuzzy PROMETHEE

Fuzzy logic and PROMETHEE are two concepts combined to form fuzzy PROMETHEE. This combination of concepts has only been explored by a minor percentage of previous studies. PROMETHEE stands for Preference Ranking Organization Method for Enrichment Evaluation. It has been shown to effectively compare alternative methods using vital materials (criteria) to determine their performance. These criteria are qualitative values that are converted into the fuzzy scale and weighted (for each criterion) to define linguistic data. The result will provide a ranking of the alternatives from the most favorable choice to the least favorable choice. Some of the earliest studies that used this methodology include [55–62].

More studies in 2019 incorporated fuzzy PROMETHEE for various medical applications. They include studies on antiretroviral combination decision in pediatric HIV therapy [46], sterilization methods for medical devices [63], postexposure prophylaxis regimen in the prevention of potential pediatric HIV-1 infection [64], and selection of most appropriate antiretroviral drugs in focused aged groups of HIV-1 infected children [64]. All of these studies made an effective comparative analysis of related alternatives in various fields depending on the necessary and important criteria and importance weights.

The article "The Efficiency of AuNPs in Cancer Cell Targeting Compared to Other Nanomedicine Technologies Using Fuzzy PROMETHEE" was published in 2021. Journal: J Healthc Eng.

The fuzzy PROMETHEE is an MCDM method that analyzes multicriteria scenario and makes a ranking organizational method for comparison and evaluation purposes [65]. Comparison for decision-making in complex issues such as anticancer drug delivery is usually difficult to achieve; however, fuzzy PROMETHEE was developed to tackle such challenges. The technique can complete the comparison process with both numerical and nonnumerical values by converting linguistic variables into mathematical variables.

Criteria are weighted according to previous literature. These weights can be altered according to the researcher's preference. Yager index was used in the defuzzification of data because it considers all the points and is not hugely affected by extreme values or weights. Lastly, defuzzified values were imputed into PROMETHEE GAIA decision lab software with Gaussian preference function (GPF) for the comparative analysis of NPs.

### 2.2. Dataset

Theranostic NPs for anticancer were selected after an extensive review of previous studies on NPs. Appropriate standards were chosen for the method of engineering and modification of NPs specifications for improved exploitation of their advantages, thus enhancing therapeutic efficiency. Furthermore, the criteria adopted included NPs manufacturing cost, size, shape, surface charge (SC), noncovalent ligand type (NCL), stimuli effects (pH and temperature), biocompatibility (BC), toxicity (TO), targeting specificity (SP), stability (ST), efficacy (EF), adverse effects (AE), and patient safety (SA). These criteria are vital for enhanced biocompatibility, encapsulation, controlled biodegradability, leakage, and circulation time in the blood; targeting the desired site efficiently with high specificity; and stability with very specific doses. NPs accumulation (ACC) in the body is significantly related to their toxicity/cytotoxicity that may cause adverse side effects. Thus, toxicity/cytotoxicity was included as an important criterion for the selection of NPs as anticancer drug carriers. Tables 1 and 2 show the dataset including selected NPs for anticancer drug delivery, criteria, and corresponding visual PROMETHEE values

A triangular fuzzy scale was utilized with weight selection for each criterion, distinguishing one criterion from another clearly and directly reflecting the order of priority. Weight was assigned to each criterion of NPs depending on the importance of the criterion. The criteria size, shape, surface charge, biocompatibility, accumulation ratio, toxicity, efficacy, adverse effects, and safety were classified within the first-degree importance, and the maximum weight was assigned as “very high” with fuzzy number ranging within (0.75, 0.92, 1.00) because of the extreme importance to improvement of drug targeting, enhanced treatment efficiency, and patient safety, thus increasing survival rate and quality life. Other criteria like pH, temperature, ligand type, specificity, and stability were assigned second-degree importance as “high” weight with fuzzy number ranging within (0.50, 0.75, 1.00) because of the indirect effect on survival rate. Finally, the cost of manufacturing is assigned the least importance on the scale “moderate” weight with fuzzy number ranging within (0.25, 0.50, 0.75), since all the previous parameters are much more important for the cure and safety of the patient compared with the latter one.  Table 3 shows linguistic variables and their corresponding priority weight of criteria and fuzzy numbers.

The article "The Efficiency of AuNPs in Cancer Cell Targeting Compared to Other Nanomedicine Technologies Using Fuzzy PROMETHEE" was published in 2021. Journal: J Healthc Eng.

## 3. Result and Discussion

The resulting order through the total net flow of the visual PROMETHEE scenario ranking illustrates the sequence of the NPs from the top to the bottom in terms of the performance of each NP as intelligent drug delivery system for anticancer treatment. The domain from the net flow point to the positive outranking flow states the cumulative performance of NPs; however, the range from the net flow point to the negative outranking flow states the descending performance. The resulting sequence shown in Table 4 indicates that AuNPs were ranked in first place with highest net flow (Phi) equal to 0.1428, positive outranking flow (+Phi) equal to 0.1428, and zero negative outranking flow (−Phi), followed by polymeric micelles with Phi = 0.0280, positive Phi = 0.0511, and negative Phi = 0.0231. The quantum dots (QDs) had Phi = −0.0467, positive Phi = 0.0225, and negative Phi = 0.0692. The dendrimers had net flow Phi = −0.0593, positive Phi = 0.0111, and negative Phi = 0.0703. Ultimately, the last place was taken by the liposomes with Phi = −0.0649, positive Phi = 0.0110, and negative Phi = 0.0759. The result provides a complete ranking of NPs from the best specific group of NPs used in the treatment of cancer to the least which is beneficial for decision-making. This considers all input factors or criteria necessary for designing intelligent anticancer drug carriers and then provides ranking.

The action profile for each NP included in this study has been illustrated and clarified according to Figure 1, and the results provide absolute strength and weaknesses of each alternative NP. AuNPs were ranked in the first place due to the classification, and its resulting action profile is all design criteria as very good modification choices starting from the size of the particle followed by the shape and thermal sensitivity, accumulation ratio with good biocompatibility, and pH sensitivity, in addition to the high ability to functionalize the AuNPs surface with noncovalent ligand and moderated surface charge performance. These decorating factors result in high percentage of biocompatibility, targeting specificity, and therapeutic efficiency with favorable stability, with no systematic toxicity or adverse effects, which guarantees the patient's safety. The polymeric micelles were assorted in the second place, and the action profile states that the main problem for the PMs is related to the shape of the PMs and the high accumulation rate resulting in systematic toxicities. The dendrimers were classified in the third place, and the action profile emphasizes that the main problem with dendrimers NPs is related to the modified size performance and the specificity of targeting, resulting in therapeutic deficiency. The unfavorable stimuli factor performance (pH) and ligand type of the dendrimers in addition to the accumulation rate of the particle in the body cause side effects and deficiency in patient safety factor. The liposomes have been rated in the fourth place, and from the action profile it is clear that the behavior of these NPs as intelligent anticancer drug delivery system suffers from serious problems in the systematic toxicity, in addition to deficiencies in the surface charge, temperature stimulus factor, and biocompatibility in one level. In the other level, there is the pH sensitivity, ligand type, particle shape, and stability. Overall, these results lead to mild liposome accumulation rate in the body, mild targeting specificity, low side effect, very low therapeutic efficiency, and patient safety.

The article "The Efficiency of AuNPs in Cancer Cell Targeting Compared to Other Nanomedicine Technologies Using Fuzzy PROMETHEE" was published in 2021. Journal: J Healthc Eng.

The quantum dots were in the last place, and from the action file the main weakness point in this type was due to the deficiency in the thermal sensitivity and the accumulation rate in the body due to the size of the particle which causes side effects and insufficient therapeutic results, in addition to other problems in pH sensitivity, ligand type, and specificity. Despite the serious problems that these atoms suffer from due to the accumulation rate, these particles are rather nontoxic and have the possibility of discharging out of the body after a while.

## 4. Conclusion

Deciding on the right technique to treat cancer with no side effects can be made using nanomedicine technologies by exploiting the advantages of both the features used and the characteristics of the cancerous environment of the infected cell which entirely differs from the healthy cell. Nanomedicine can enhance therapeutic effectiveness of cancer treatment techniques to a new level of efficiency and patient's safety and reduce the chances of secondary infection as side effects of treatment.

The article "The Efficiency of AuNPs in Cancer Cell Targeting Compared to Other Nanomedicine Technologies Using Fuzzy PROMETHEE" was published in 2021. Journal: J Healthc Eng.

This study used fuzzy PROMETHEE that employs double comparison in fuzzy conditions. It discussed a set of important specifications for a group of nanoparticles that are considered as ideal options for designing intelligent systems to deliver anticancer drugs, against set of designing criteria. Each criterion in turn was given an importance factor. The outcomes of the study indicate that AuNPs are determined as preferred alternatives, while PMs, QDs, dendrimers, and liposomes are less preferred alternatives, respectively. The criteria that were selected for determining AuNPs showed high effectiveness of loading and delivering the drug to the targeted cell with almost no side effects. The proposed method is capable of merging qualitative and quantitative data, which makes it unique. Its efficacy and ease of use make it one of the best methods of visualization and application compared to the other MCDM methods. It is also very applicable to and suitable for creating a knowledge-based system of design.

## Figures and Tables

**Figure 1:** PROMETHEE rainbow showing a complete ranking and action profile of the selected NPs from the specific group of NPs used in the treatment of cancer to the least.

**Table 1:** Nanoparticles used as anticancer drug delivery vehicles, their respective parameters, and their corresponding visual PROMETHEE values.

Criteria	Cost	Size	Shape	pH	Temp	SC	NCL
Unit	($)	(nm)			(C)		
*Preference*							
Max\min	Min	Max	Max	Max	Max	Max	Yes
Weight	M	VH	VH	H	H	VH	H
Preference fn.	Gaussian	Gaussian	Gaussian	Gaussian	Gaussian	Gaussian	Gaussian

*Evaluation*							
AuNPs	M	VG	VH	VG	VH	VG	Yes
Liposomes	VH	A	M	G	M	A	No
Dendrimers	H	G	M	G	H	A	No
PMs	H	A	H	G	M	G	No
QDs	M	G	H	G	VH	G	No

^∗^AuNPs: gold nanoparticles; PMs: polymeric micelles; QDs: quantum dots; Temp: thermal conductivity; SC: surface charge; NCL: noncovalent legend; H: high; M: medium; VH: very high; A: average; G: good; VG: very good.

**Table 2:** Nanoparticles used as anticancer drug delivery vehicles, their respective parameters, and their corresponding visual PROMETHEE values.

Criteria	BC	ACC	TO	SP	ST	EF	AE	SA
Unit	%	%	%	%	%	%	%	%

*Preference*								
Max\min	Max	Min	Min	Max	Max	Max	Min	Max
Weight	VH	VH	VH	H	H	VH	VH	VH
Preference fn.	Gaussian	Gaussian	Gaussian	Gaussian	Gaussian	Gaussian	Gaussian	Gaussian

*Evaluation*								
AuNPs	VH	VL	VL	VH	VH	VH	VL	VH
Liposomes	H	H	H	H	H	H	L	L
Dendrimers	M	H	M	M	M	M	M	M
PMs	H	M	M	H	H	VH	L	H
QDs	M	H	L	H	M	H	H	VL

^∗^AuNPs: gold nanoparticles; PMs: polymeric micelles; QDs: quantum dots; BC: biocompatibility; ACC: accumulation rate; TO: toxicity; SP: specificity; ST: stability; EF: efficacy; AE: adverse effect; SA: safety; H: high; M: medium; VH: very high; L: low; VL: very low; A: average; G: good; VG: very good.

The article "The Efficiency of AuNPs in Cancer Cell Targeting Compared to Other Nanomedicine Technologies Using Fuzzy PROMETHEE" was published in 2021. Journal: J Healthc Eng.

**Table 3:** Linguistic variables and their corresponding priority weight of criteria and fuzzy numbers.

Priority weight of criteria	Fuzzy number	Rating of criteria
Very high (VH)	(0.75, 1.00, 1.00)	Size, shape, surface charge, biocompatibility, accumulation ratio, toxicity, efficacy, adverse effect, safety
High (H)	(0.50, 0.75, 1.00)	pH, temperature, noncovalent ligand, specificity, stability
Moderate (M)	(0.25, 0.50, 0.75)	Cost
Low (L)	(0, 0.25, 0.50)	
Very low (VL)	(0, 0, 0.25)	

**Table 4:** A complete ranking of nanoparticles as anticancer drug delivery.

Rank	Nanoparticles as intelligent anticancer drug delivery	Phi	Phi+	Phi−
1	AuNPs	0.1428	0.1428	0.0000
2	Polymeric micelles	0.0280	0.0511	0.0231
3	Quantum dots	−0.0467	0.0225	0.0692
4	Dendrimers	−0.0593	0.0111	0.0703
5	Liposomes	−0.0649	0.0110	0.0759

## Data Availability

The data used and/or analyzed during the current study is already available from the literature.

## References

[1] Mundasad S. (2018). Cancers rising around the world. https://www.bbc.com/news/health-45497304.

[2] Siegel R. L., Miller K. D., Jemal A. (2019). Cancer statistics.

[3] Who (2018). Cancer; key facts. https://www.who.int/news-room/fact-sheets/detail/cancer.

[4] Bahrami B., Hojjat-Farsangi M., Mohammadi H. (2017). Nanoparticles and targeted drug delivery in cancer therapy. *Immunology Letters*.

[5] Bhatia S., Bhatia S. (2016). Nanoparticles types, classification, characterization, fabrication methods and drug delivery applications, 33-93. *Natural Polymer Drug Delivery Systems*.

[6] Fragouli P. G., Stavroulaki D., Christakopoulos P., Makhlouf A. H., Abu-Thabit N. Y. (2019). Responsive polymeric micelles for drug delivery applications/cancer. *Stimuli Responsive Polymeric Nanocarriers for Drug Delivery Applications, Volume 2: Advanced Nanocarriers for Therapeutics. A Volume in Woodhead Publishing Series in Biomaterials*.

[7] Sneider A., VanDyke D., Paliwal S., Rai P. (2017). Remotely triggered nano-theranostics for cancer applications. *Nanotheranostics*.

[8] Li Z., Tan S., Li S., Shen Q., Wang K. (2017). Cancer drug delivery in the nano era: an overview and perspectives (Review). *Oncology Reports*.

[9] Albanese A., Tang P. S., Chan W. C. (2012). The effect of nanoparticle size, shape, and surface chemistry on biological systems. *Annual Review of Biomedical Engineering*.

[10] Shen Z. H., Nieh M. P., Li Y. (2016). Decorating nanoparticle surface for targeted drug delivery: opportunities and challenges. *Polymers*.

The article "The Efficiency of AuNPs in Cancer Cell Targeting Compared to Other Nanomedicine Technologies Using Fuzzy PROMETHEE" was published in 2021. Journal: J Healthc Eng.

[11] Poon Z., Chang D., Zhao X., Hammond P. T. (2011). Layer-by-layer nanoparticles with a pH-sheddable layer for in vivo targeting of tumor hypoxia. *ACS Nano*.

[12] Kong F., Zhang J., Li R., Wang Z., Wang W., Wang W. (2017). Unique roles of gold nanoparticles in drug delivery, targeting and imaging applications. *Molecules*.

[13] Hainfeld J. F., Slatkin D. N., Focella T. M. (2005). Gold nanoparticles: a new X-ray contrast agent. *British Journal of Radiology*.

[14] Fratoddi I., Venditti I., Cametti C., Russo M. V. (2015). How toxic are gold nanoparticles? The state-of-the-art. *Nano. Research*.

[15] Conde J., Doria G., Baptista P. (2012). Noble metal nanoparticles applications in cancer. *Journal of Drug Delivery*.

[16] Cho K., Wang X., Nie S., Zhuo N., Dong C., Shin M. (2008). Therapeutic nanoparticles for drug delivery in cancer. American association for cancer research. *Clinical Cancer Research*.

[17] Senapati S., Mahanta A. K., Kumar S., Maiti P (2018). Controlled drug delivery vehicles for cancer treatment and their performance. *Signal Transduction Targeted Therapy*.

[18] Hossen S., Khalid H. M., Basher M. K., Mia M.N.H., Rahman M.T., Uddin M. J. (2019). Smart nanocarrier-based drug delivery systems for cancer therapy and toxicity studies: a review. *Journal of Advertising Research.*.

[19] Elahi N., Kamali M., Baghersad M. H. (2018). Recent biomedical applications of gold nanoparticles: a review. *Talanta*.

[20] Chompoosor A., Han G., Rotello V. M. (2008). Charge dependence of ligand release and monolayer stability of gold nanoparticles by biogenic thiols. *Bioconjugate Chemistry*.

[21] Kim Y., Johnson R. C., Hupp J. T. (2001). Gold nanoparticle-based sensing of “spectroscopically silent” heavy metal ions. *Nano Letters*.

[22] Liu C. W., Hsieh Y. T., Huang C. C., Lin Z. H., Chang H. T. (2008). Detection of mercury(II) based on Hg2+-DNA complexes inducing the aggregation of gold nanoparticles. *Chemical Communications*.

[23] Wilson G. S., Hu Y. B. (2000). Enzyme based biosensors for in vivo measurements. *Chemical Reviews*.

[24] Zhang S. X., Wang N., Yu H. J., Niu Y. M., Sun C. Q. (2005). Covalent attachment of glucose oxidase to an Au electrode modified with gold nanoparticles for use as glucose biosensor. *Bioelectrochemistry*.

[25] Jin L. H., Shang L., Guo S. J. (2011). Biomolecule-stabilized Au nanoclusters as a fluorescence probe for sensitive detection of glucose. *Biosensors and Bioelectronics*.

[26] Wen F., Dong Y. H., Feng L., Wang S., Zhang S. C., Zhang X. R. (2011). Horseradish peroxidase functionalized fluorescent gold nanoclusters for hydrogen peroxide sensing. *Analytical Chemistry*.

[27] Crespilho F. N., Ghica M. E., Florescu M., Nart F. C., Oliveira O. N., Brett C. M. A. (2006). A strategy for enzyme immobilization on layer-by-layer dendrimer-gold nanoparticle electrocatalytic membrane incorporating redox mediator. *Electrochemistry Communications*.

The article "The Efficiency of AuNPs in Cancer Cell Targeting Compared to Other Nanomedicine Technologies Using Fuzzy PROMETHEE" was published in 2021. Journal: J Healthc Eng.

[28] Lia Y., Schluesenerb H. J., Xu S. (2010). Gold nanoparticle-based biosensors. *Gold Bulletin*.

[29] Yehezkeli O., Vered R. T., Raichlin S., Willner I. (2011). Nano-engineered flavin-dependent glucose dehydrogenase/gold nanoparticle-modified electrodes for glucose sensing and biofuel cell applications. *ACS Nano*.

[30] Holland J. T., Lau C., Brozik S., Atanassov P., Banta S. (2011). Engineering of glucose oxidase for direct electron transfer via site-specific gold nanoparticle conjugation. *Journal of the American Chemical Society*.

[31] Wu Z., Jin R. (2010). On the ligand’s role in the fluorescence of gold nanoclusters. *Nano Letters*.

[32] Yoo C. I., Seo D., Chung B. H., Chung I. K., Song H. (2009). A facile one-pot synthesis of hydroxyl-functionalized gold polyhedrons by a surface regulating copolymer. *Chemistry of Materials*.

[33] Shem P. M., Sardar R., Shumaker-Parry J. S. (2009). One-step synthesis of phosphine-stabilized gold nanoparticles using the mild reducing agent 9-BBN. *Langmuir*.

[34] Ding Y., Zhang X., Liu X., Guo R. (2006). Adsorption characteristics of thionine on gold nanoparticles. *Langmuir*.

[35] Khanna S. C., Jecklin T., Speiser P. (1970). Bead polymerization technique for sustained-release dosage form. *Journal of Pharmacological Sciences*.

[36] Noble G. T., Stefanick J. F., Ashley J. D., Kiziltepe T., Bilgicer B. (2014). Ligand-targeted liposome design: challenges and fundamental considerations. *Trends in Biotechnology*.

[37] Lee Y., Thompson D. H. (2017). Stimuli-responsive liposomes for drug delivery. *Wiley Interdiscip Rev. Nanomed. Nanobiotech.*.

[38] Petersen A. L., Hansen A. E., Gabizon A., Andresen T. L. (2012). Liposome imaging agents in personalized medicine. *Advanced Drug Delivery Reviews*.

[39] Vahed Z. S., Salehi R., Davaran S., Sharifi S. (2017). Liposome-based drug co-delivery systems in cancer cells. *Materials Science and Engineering: C*.

[40] Buhleier E., Wehner W., Vögtle F. (1978). ‘Cascade’- and ‘nonskidchain- like’ syntheses of molecular cavity topologies. *Synthesis-stuttgart (Mass)*.

[41] Jackson C. L., Chanzy H. D., Booy F. P. (1998). Visualization of dendrimer molecules by transmission electron microscopy (TEM): staining methods and cryo-TEM of vitrified solutions. *Macromolecules*.

[42] Khopade A. J., Caruso F., Tripathi P., Nagaich S., Jain N. K. (2002). Effect of dendrimer on entrapment and release of bioactive from liposomes. *International Journal of Pharmacy*.

The article "The Efficiency of AuNPs in Cancer Cell Targeting Compared to Other Nanomedicine Technologies Using Fuzzy PROMETHEE" was published in 2021. Journal: J Healthc Eng.

[43] Tao X., Yang Y. J., Liu S., Zheng Y. Z., Fu J., Chen J. F. (2013). Poly (amidoamine) dendrimer-grafted porous hollow silica nanoparticles for enhanced intracellular photodynamic therapy. *Acta Biomaterialia*.

[44] Quintana A., Raczka E., Piehler L. (2002). Design and function of a dendrimer-based therapeutic nanodevice targeted to tumor cells through the folate receptor. *Pharmaceutical Research*.

[45] Kutuzov S., He J., Tangirala R., Emrick T., Russell T. P., Böker A. (2007). On the kinetics of nanoparticle self-assembly at liquid/liquid interfaces. *Physical Chemistry Chemical Physics*.

[46] Mukerjee P., Chan C. C. (2002). Effects of high salt concentrations on the micellization of octyl glucoside: salting-out of monomers and electrolyte effects on the micelle–water Interfacial tension. *Langmuir*.

[47] Quinn B. M., Liljeroth P., Ruiz V., Laaksonen T., Kontturi K. (2003). Electrochemical resolution of 15 oxidation states for monolayer protected gold nanoparticles. *Journal of the American Chemical Society*.

[48] Croy S. R., Kwon G. S. (2006). Polymeric micelles for drug delivery. *Current Pharmaceutical Design*.

[49] Sutton D., Nasongkla N., Blanco E., Gao J. (2007). Functionalized micellar systems for cancer targeted drug delivery. *Pharmaceutical Research*.

[50] Cajot S., Schol D., Danhier F., Préat V., Gillet De Pauw M. C., Jérôme C. (2013). In vitro investigations of smart drug delivery systems based on redox-sensitive cross-linked micelles. *Macromolecular Bioscience*.

[51] Husseini G. A., Runyan C. M., Pitt W. G. (2002). Investigating the mechanism of acoustically activated uptake of drugs from Pluronic micelles. *BMC Cancer*.

[52] Seo S. J., Lee S. Y., Choi S. J., Kim H. W. (2015). Tumor-targeting Co-delivery of drug and gene from temperature-triggered micelles. *Macromolecular Bioscience*.

[53] Bailey R. E., Smith A. M., Nie S. (2004). Quantum dots in biology and medicine. *The Physical Educator*.

[54] Gao X., Cui Y., Levenson R. M. (2004). In-vivo cancer targeting and imaging with semiconductor quantum dots. *Nature Biotechnology*.

[55] Gokcekus H., Ozsahin D., Mustapha M. (2020). Simulation and evaluation of water sterilization devices. *Desalination and water treatment*.

[56] Ozsahin D., Gelisen M., Mustapha M., Agachan Y., Rahi D., Uzun B. (2021). Decision analysis of the COVID-19 vaccines. *The EuroBiotech Journal*.

[57] Mustapha M., Uzun B., Uzun Ozsahin D., Ozsahin I. (2021). A comparative study of X-ray based medical imaging devices. *Applications of Multi-Criteria Decision-Making Theories in Healthcare and Biomedical Engineering*.

[58] Mustapha M., Uzun Ozsahin D., Ozsahin I. (2021). Comparative evaluation of point-of-care glucometer devices in the management of diabetes mellitus. *Applications of Multi-Criteria Decision-Making Theories in Healthcare and Biomedical Engineering*.

The article "The Efficiency of AuNPs in Cancer Cell Targeting Compared to Other Nanomedicine Technologies Using Fuzzy PROMETHEE" was published in 2021. Journal: J Healthc Eng.

[59] Ozsahin D. U., Uzuna B., Musaa M. S., Şentürka N., Nurçina F. V., Ozsahina I. (2017). Evaluating nuclear medicine imaging devices using fuzzy PROMETHEE method. *Procedia Computer Science*.

[60] Uzun O. D., Isa N. A., Uzun B., Ozsahin I. Effective analysis of image reconstruction algorithms in nuclear medicine using fuzzy PROMETHEE.

[61] Uzun B., Sultanoğlu N., Sayan M., Sanlidag T., Ozsahin D. U. Selection of the most appropriate antiretroviral medication in determined aged groups (≥3 years) of HIV-1 infected children.

[62] Ozsahin I., Mustapha M. T., Albarwary S., Sanlidag B, Ozsahin D. U., Butler T. A. (2021). An investigation to choose the proper therapy technique in the management of autism spectrum disorder. *Journal of Comparative Effeactivenes Research*.

[63] Taiwo M. M., Ozsahin I., Ozsahin D. U. Evaluation of sterilization methods for medical devices.

[64] Sayan M., Sultanoğlu N., Sarıgul F., Sanlidag T., Ozsahin D. U. Determination of post-exposure Prophylaxis regimen in the prevention of potential pediatric HIV-1 infection by the multi-criteria decision-making theory.

[65] Brans J. P., Vincke P. H., Mareschal B. (1986). How to select and how to rank projects: the PROMETHEE method. *European Journal of Operational Research*.

